The article "Effect of Aeolian Sand Powder Addition on Frost Resistance of Concrete Pavement" was retracted in 2023. Reasons: signs of a paper mill; suspected computer-generated content; unreliable results or conclusions; concerns about the data.

# Effect of Aeolian Sand Powder Addition on Frost Resistance of Concrete Pavement

**DOI:** 10.1155/2022/5087896

**Published:** 2022-07-04

**Authors:** Ou Zhao, Xuefeng Deng

**Affiliations:** Hunan Urban Construction College, Xiangtan, Hunan, 411101, China

## Abstract

In order to solve the problem of exploring the freeze-thaw characteristics of modified aeolian sand mixed with cement and silt, the authors propose a freeze-thaw cycle test of modified aeolian sand under the condition of mixing 5% cement and silt with different contents. In this experiment, under freeze-thaw conditions, its intensity decay and mass volume change law and the changes of freeze-thaw characteristics were comprehensively characterized by multiple indicators. The result shows that, after two freeze-thaw cycles, the compressive strength and peak strain of the improved aeolian sand were positively correlated with the silt content. With the increase of the number of freeze-thaw cycles, the compressive and antidestruction capacity of the improved aeolian sand with high silt content and low silt content decreased significantly. 15% silt content improves the structural stability of aeolian sand. It is proved that the authors' experiment can intuitively and effectively reflect the change law of soil strength after freezing and thawing of such improved aeolian sandy soil, which has displayed significance.

## 1. Introduction

Cement is one of the three main materials, and it has an irreplaceable position in the current construction industry [1]. With the rapid development of infrastructure and real estate in our country, the demand for cement is also increasing. At the same time, the pollution problem is also very serious, especially in the cement production process, as the emission and noise of dust and CO_2_ have caused great harm to the human living environment [2]. Therefore, it is of great significance to find some low-energy consumption admixtures to replace part of the cement. It can not only solve the environmental harm caused by the accumulation of solid waste but also add admixtures to concrete to delay the early hydration of cement and avoid the heat of hydration. Excessive damage has a positive effect on the strength and durability of concrete in the later stage [3] as shown in Figure 1.

Aeolian sand, also known as desert sand, is a siliceous material that is naturally transported to alluvial plains by wind and is widely distributed in Xinjiang, Inner Mongolia, and other places in China [4]. In recent years, desertification and sandification in China have become more and more serious, the area of desertified land is about 2.62 million square kilometers, and the area of desertified land is about 1.73 million square kilometers. In wind and sand eroded roads, and during spring, sand and dust are all over the sky, so the ecological environment is seriously damaged [5]. With the implementation of the country's western development strategy, the consumption of concrete is increasing day by day. In Inner Mongolia, river sand resources are scarce, aeolian sand reserves are abundant, and the rational development and utilization of aeolian sand resources is one of the most effective ways to solve these problems [6].

The article "Effect of Aeolian Sand Powder Addition on Frost Resistance of Concrete Pavement" was retracted in 2023. Reasons: signs of a paper mill; suspected computer-generated content; unreliable results or conclusions; concerns about the data.

Seasonally frozen areas in China are widely distributed. The problems of soil strength and deformation caused by freeze-thaw cycles are very common, and the prevention and control of freezing damage has become the focus of long-term engineering attention [7]. Northwest seasonally frozen areas such as Gansu and other places are adjacent to the Tengger Desert, where a large range of aeolian sand is distributed, which has the characteristics of single particle size and poor particle cohesion, and it is difficult to directly use it as a building material [8]. However, the construction of civil and water conservancy projects in the abovementioned areas often has to use aeolian sand as a building material. Therefore, the treatment and resource utilization of aeolian sand in seasonally frozen areas is of great engineering significance.

## 2. Literature Review

Due to the loose accumulation of aeolian sand, the content of silty clay is low and cannot store water, so it is difficult for vegetation to survive. In addition to the influence of wind, aeolian sand will expand infinitely with the direction of the wind, swallowing the original land resources, and this results in the reduction of arable land and livestock areas, which seriously threatens the survival of human beings [9]. Every spring, yellow sand fills the sky, the air is turbid, dust and sandstorms often occur, and the dust content in the air far exceeds the national regulations, which not only causes respiratory diseases but also affects travel safety. Therefore, the problem of desertification requires urgent need of treatment [10]. Many scholars at home and abroad have carried out applied research on it. By studying the effect of adding extra-fine sand in concrete on the workability of the mixture, the pumping of ultrafine sand concrete is realized [11]. The aeolian sand mortar is configured by replacing the river sand by the internal mixing method, etc., and it was found that when 20% of the river sand was replaced, the fluidity of the mortar and strength were improved [12].

The common aeolian sand resource utilization improvement technology is the single-mixed cement modification method, Yong-long studied the factors affecting the unconfined compressive strength of cement-modified aeolian sand through laboratory experiments. It was found that the strength of the improved soil was positively correlated with the curing age, compaction coefficient, and cement strength grade [13]. Liu explored and found that, under the action of salt-freeze coupling, the unconfined compressive strength and pore volume of cement-modified aeolian sand showed a negative linear law, and the elastic modulus decreased with the increase of freeze-thaw times [14]. Chen studied the effect of cement content on the strength and deformation characteristics of aeolian sand foundation and believed that there is an optimal ratio between the natural moisture content of aeolian sand and cement content, which can significantly improve the strength and deformation performance of the original soil [15]. As can be seen, the principle of cement to improve this kind of soil is to generate cementitious substances such as calcium silicate hydrate, in order to enhance the curing and bonding effect [16]. Considering the economy, there are also other admixture improvement studies, such as Wang Research, on the effect of cohesive soil on the uniaxial compressive strength of aeolian sand under the conditions of different freeze-thaw times. It is believed that the essence of strength improvement is that the clay particles bind the water film to make the sand particles bond more tightly [17]. Zhang Y. found that an appropriate amount of silty clay can fill the pores between the sand grains, the overall compactness is improved, but the addition of too much powder and clay will lead to a decrease in the strength index [18]. Wang studied the technology of improving aeolian sand with fine round gravel soil and inorganic cementitious materials, respectively, and believed that such external admixtures could improve the gradation of aeolian sand and improve soil compactness. However, the freeze-thaw characteristics of the improved soil were not mentioned [19]. In summary, at present, most studies on the mechanical properties of aeolian sand after freeze-thaw cycles are limited to the effects of single-mixed cement or silt, and there is no report on the freeze-thaw performance of improved aeolian sand mixed with cement and silt.

The article "Effect of Aeolian Sand Powder Addition on Frost Resistance of Concrete Pavement" was retracted in 2023. Reasons: signs of a paper mill; suspected computer-generated content; unreliable results or conclusions; concerns about the data.

On the basis of the current research, the authors studied the effect of different mixing ratios and different freeze-thaw cycles, variation law of unconfined compressive strength, and failure strain and elastic modulus of improved aeolian sandy soil. The mass loss and volume change of the improved soil under various mixing ratios were quantitatively analyzed, and the optimal mixing ratio and strength change mechanism of the mixed improved sandy soil were analyzed, in order to provide a basis for the application of engineering technology.

## 3. Research Methods

### 3.1. Test Materials

The aeolian sand used in the test was taken from the field area outside a reservoir. Due to the long-term wind erosion in the field, the particle size of the aeolian sand is relatively fine, and its main components are quartz, debris, and feldspar. *d*_10_ = 0.080 mm, *d*_30_ = 0.097 mm, *d*_60_ = 0.138 mm, *C*_u_ = 1.725, and *C*_c_ = 0.852. It is a poorly graded sandy soil [20].

The cement used in the test is Conch brand ordinary Portland cement P•O 42.5. Because the test area is located in an alluvial plain, the upper soil layer is rich in silty loam resources, which can provide a source of silt for this test [21].

### 3.2. Selection of Cement and Silt Content

According to GBT50123–2019 “Geotechnical Test Method Standard,” the dry density index and relative density of modified aeolian sand samples with a single cement content of 0. 3%, 5%, and 7% were obtained, respectively, and the results are shown in Table 1 [22].

According to the relevant local design and construction safety requirements, when the compaction degree of the filling is 96%, the relative density should be guaranteed to be greater than 0.80 [23]. Therefore, adding 5% cement to improve aeolian sand meets the requirements of the relative density index, and it is more economical than adding 7% cement [24]. Therefore, the authors chose 5% cement content as the modified cement content in the experiment.

The particle size of aeolian sand is relatively single, and the cohesion between particles is low. For general economic considerations, the method of adding 5% cement alone can only improve the bonding between sand particles, and the overall compaction effect is not obvious; Mixing appropriate amount of silt and cement, without changing the cohesion between particles, significantly improved pore filling compactness [25]. Considering the same external work conditions, the compacted dry density can reflect the compaction effect of mixing and filling of such materials, in order to select a reasonable amount of silt for improvement. The authors conducted a standard compaction test of 3%–20% silt alone.

If the content of single-mixed silt exceeds 9%, it can significantly increase the dry density. Considering the economy, the dosage threshold for single-mixed silt to achieve the best compaction effect is 15%–20%, and the increase of maximum dry density of silty soil mixed with 15%-20% is about half of that with 13%-15%. Silt content exceeds 20%, and the compaction effect is not significant. Therefore, in order to explore the freeze-thaw degradation characteristics of modified aeolian sand with different silt contents under the economical cement content of 5%, four groups of silt contents were selected in the experiment: 5% cement + 0% silt (baseline), 5% cement + 10% silt, 5% cement + 15% silt, and 5% cement + 20% silt.

The article "Effect of Aeolian Sand Powder Addition on Frost Resistance of Concrete Pavement" was retracted in 2023. Reasons: signs of a paper mill; suspected computer-generated content; unreliable results or conclusions; concerns about the data.

### 3.3. Sample Preparation

The tests are divided into macroscopic tests of freeze-thaw cycles, unconfined compression, mass loss, and volume change rate.

According to the “Standards for Geotechnical Test Methods,” standard heavy-duty compaction tests were carried out on the above four groups of modified aeolian sandy soils, respectively, and the maximum dry density and optimum moisture content of each group of samples were obtained. Considering that the different compaction degree and moisture content of the samples will affect the results of the freeze-thaw cycle, all soil samples were controlled according to the standard of 96% compaction degree under the optimal moisture content condition, and the samples were compacted and prepared in 5 layers. The standard size of the cylinder sample is diameter *D* = 61.8 mm and height *H* = 125 mm.

The clay content in this kind of aeolian sand improved mixed soil is relatively low, and the soil particles are weakly bonded, and there is certain randomness. In order to obtain reliable test rules, this test was based on six freeze-thaw cycles from 0 to 12 times as the loading standard, three parallel samples were set under each working condition, and a total of 84 samples were produced. During sample preparation, make sure that the compaction is completed within the initial setting time of the cement. In order to avoid moisture loss, the samples taken out from the layered sample preparation cylinder should be wrapped with plastic wrap immediately, and the curing room was maintained for 14 days.

### 3.4. Evaluation Indicators

Freeze-thaw test uses a HDD-II freeze-thaw tester and UTM4503 electronic universal tester. The control accuracy can reach ±0.1°C, and each freeze-thaw cycle is divided into 4 stages: cooling section (4 h), low temperature holding section (3 h), heating section (4 h), and high temperature holding section (3 h), in which the low temperature is −20°C and the high temperature is 20°C, a total of 12 cycles. The electronic universal testing machine adopts strain loading control, the rate control is 1.25 mm/min, and the loading of the sample is stopped when the cumulative 20% strain is loaded. In addition, in order to reduce the end effect during the compression process of the sample, a thin layer of vantulin was applied to the loading surface of the sample before the test.

The article "Effect of Aeolian Sand Powder Addition on Frost Resistance of Concrete Pavement" was retracted in 2023. Reasons: signs of a paper mill; suspected computer-generated content; unreliable results or conclusions; concerns about the data.

The volume change rate was measured with a 0.01 mm high-precision vernier caliper to measure the diameter and height of the soil sample in the freezing and thawing state, and the average height in the orthogonal direction was taken. A single sample was divided into 5 layers to measure the diameter, the average value was obtained, and the sample volume was obtained after deducting the thickness of the plastic wrap. The mass loss rate and volume change rate are, respectively,

(1) $$\begin{array}{c} \delta_{m}=\frac{M_{0}-M_{N}}{M_{0}}\times 100\%, \end{array}$$

(2) $$\begin{array}{c} \varepsilon_{m}=\frac{V_{N}-V_{0}}{V_{0}}\times 100\%. \end{array}$$

In the formula, *M*_*N*_ and *V*_*N*_ are the mass and volume of the sample after *N* freezing and thawing, after deducting the plastic wrap.

## 4. Analysis of Results

### 4.1. Stress-Strain Relationship

During the freeze-thaw cycle, in addition to the microscopic water phase transition, it is also accompanied by mesoscopic random particle exfoliation and structural reorganization. Due to the low internal cohesion of the modified aeolian sand, brittle failure will occur, so the unconfined compressive stress-strain curve has random fluctuations. For this purpose, 0 (reference sample), 1, 2, and 8 freeze-thaw cycle test data were selected for analysis, as shown in Figures 2, 3(a), and 3(b).

Under uniaxial pressure loading, the soil failure experienced a compaction stage, a linear elastic stage, a nonlinear strengthening stage and a softening stage. As can be seen from Figure 2, the stress and strain of the samples with different silt contents before and after freezing and thawing are all in the strain softening failure mode, indicating that freezing and thawing will not change the failure mode of such improved soils. Without freezing and thawing, the peak stress and failure strain of different mixed samples were positively correlated with the silt content. The reason is the silt filling the pores strengthens the binding force between the sand particles. In addition, the test shows that when the silt content exceeds 15%, the compaction section of the sample is not as good as the compaction section of the sample with a silt content of 10% and below, and it shows that adding more than 15% silt can achieve better pore compaction effect.

In view of the fact that the initial freeze-thaw also has an overconsolidation “compacting effect” on such reconstituted soils, the test also showed that the initial 1-2 freeze-thaw times, compared with the non-freeze-thaw time, and the characteristics of the compaction stage of the samples with different dosages are not obvious. Similarly, after 1 or 2 freeze-thaw times, the peak stress and failure strain of samples with different silt contents decreased significantly compared with those of unfreeze-thaw samples, and the brittle failure was more significant, but it showed a positive correlation with the silt content. The reason is that the void ratio of the sample decreases due to the “compacting effect” after the initial freeze-thaw, and the failure strain decreases during the compression process, resulting in an increase in brittleness as shown in Figure 3(a). After 8 freeze-thaw cycles, the softening stage in the stress-strain curve tends to be “steep” (as shown in Figure 3(b)) because after the specimen is loaded to reach the stress peak, cracks are formed rapidly and brittle failure occurs.

The article "Effect of Aeolian Sand Powder Addition on Frost Resistance of Concrete Pavement" was retracted in 2023. Reasons: signs of a paper mill; suspected computer-generated content; unreliable results or conclusions; concerns about the data.

### 4.2. Unconfined Compressive Strength

Statistical variation of the unconfined compressive strength of the improved aeolian sand samples with the number of freeze-thaw cycles and silt content is shown in Figures 4(a) and 4(b).

Figure 4(a) shows that, with the increase of freeze-thaw times to 8, the unconfined compressive strength of the improved soil with 5% cement + 15% silt content increased, while the rest of the silt content improved soil showed a downward trend. It is also found that, during the first 8 freeze-thaw cycles, the strength attenuation of 10% silt was about 50 kPa, which was only 37% of that of 20% silt. It shows that the strength weakening factor of “part of the particle gaps, not filled” has less influence on the strength reduction than “the weakening of cement hydration and the compression of excess silt particles.”

From Figure 4(b), it can be found that except for one freeze-thaw strength abnormality (the initial structure is unstable), under the accumulative 12 freeze-thaw cycles, with the increase of silt content, the unconfined compressive strength of the improved soil showed an overall upward trend, but 15% silt. The dosage is the most significant.

Therefore, 15% silt content should be the ideal aeolian sand content improvement range.

### 4.3. Intensity Decay Law

Using the strength attenuation coefficient *S*_0_/*S*_*N*_ to analyze the variation law of the strength of the aeolian sand improved soil with four mixing ratios, Figure 5 describes the case of four doping ratios, and the ratio of the unconfined compressive strength *S*_0_ of the reference sample at 0 freeze-thaw times to the sample strength *S*_*N*_ after N freeze-thaw times changes with the number of freeze-thaw cycles.

Figure 5 also shows that except for the mixing ratio of 5% cement + 15% silt, the strength attenuation coefficient lines of the improved soils under the other three mixing ratios are as follows: the trend of rising first, then slowly rising and falling, and 5% cement + 0% silt and 5% cement + 20% silt compared with 5% cement + 10% silt. The ascending section is more “steep,” and the improved soil with high and low silt content has more obvious freeze-thaw damage when the freeze-thaw cycle is less (three times).

The article "Effect of Aeolian Sand Powder Addition on Frost Resistance of Concrete Pavement" was retracted in 2023. Reasons: signs of a paper mill; suspected computer-generated content; unreliable results or conclusions; concerns about the data.

According to the preliminary fitting regression results (5% cement + 15% silt has the most obvious fitting effect compared with other dosages), the distribution of test points at this dosage showed a great correlation with the power function *S*_0_/*S*_*N*_=1.33323*N*^−0.15728^, *R*^2^=0.97.

### 4.4. Failure Strain Characteristics

The failure strain is the strain value corresponding to the peak stress (unconfined compressive strength), which is an important indicator to describe the brittleness and plasticity of materials. At the same time, it is also an important parameter to evaluate the unconfined compression deformation characteristics of soil after freezing and thawing. Figures 6(a), 6(b) show the change law of failure strain of the improved aeolian sand sample with the number of freeze-thaw cycles and silt content.

Figure 6(a) shows that, with the increase in the number of freeze-thaw cycles, the failure strain of the improved soil with different silt contents generally increased first and then decreased.  Figure 6(b) reflects the change of failure strain with silt content. It can be seen that, before 5 times of freezing and thawing, the failure strain increased with the increase of silt content, the brittleness of the soil sample was weakened, and the toughness was improved. After 8 times of freezing and thawing, when the content of silt is less than 10%, the failure strain becomes larger. When the silt content is 10%–15%, the failure strain has a decreasing trend. When the silt content is 15%–20%, the failure strain decreases sharply, that is, after 8 freeze-thaw times, the increase of silt content and freeze-thaw times together aggravated the brittle failure of the sample.

## 5. Conclusion

The authors incorporate different contents of aeolian sand and silt into concrete and multiple temperature changes. The effect of silt content on its dynamic capacity characteristics was studied. The result obtained is as follows:

1. Based on 5% cement content as the modification benchmark, the authors experimentally studied the improvement effect of the mechanical properties of aeolian sand mixed with different silts. The result shows that freeze-thaw action does not change the brittle failure mode of unconfined compression of cement-mixed silt-modified aeolian sand. Appropriate silt content can effectively fill the pores and enhance the binding force between sand particles. Mixing 5% cement + 15% silt can achieve the effect of pore compaction.
2. During 1-2 freeze-thaw cycles, the compressive strength and peak strain of the improved aeolian sand were positively correlated with the silt content. With the increase of freeze-thaw times, the compressive and antidestruction capacities of the modified aeolian sand with high silt content and low silt content decreased significantly. The silt content of 15% improves the compactness of the aeolian sand particles, the soil compressibility is low, the stiffness is high, and the structural stability is the strongest.
3. Under freeze-thaw conditions, the volume change rate of aeolian sand mixed with cement alone and cement silt showed a downward trend on the whole, and the decrease in the content of 5% cement + 15% silt was the lowest. In view of the frost-heaving sensitive characteristics of silt, the mixed sample has a slight frost heave phenomenon (*ε* expansion ≈ 0.2*ε* shrinkage) in the local freeze-thaw cycle (4–7 times), but the single-mixed cement sample has no such phenomenon. The mass loss rate of aeolian sand improved with 5% cement alone increases linearly with the number of freeze-thaw cycles. The freezing and thawing surface spalling phenomenon of the mixed modified aeolian sand was significantly improved. After 12 freeze-thaw cycles, the change of the mass loss rate remained within 0.1%.

The article "Effect of Aeolian Sand Powder Addition on Frost Resistance of Concrete Pavement" was retracted in 2023. Reasons: signs of a paper mill; suspected computer-generated content; unreliable results or conclusions; concerns about the data.

## Figures and Tables

**Figure 1:** Frost resistance of concrete pavement.

**Figure 2:** Stress-strain law of benchmark and 1 freeze-thaw cycle.

**Figure 3:** (a) Stress-strain law under different freeze-thaw cycles. (b) Stress-strain law under different freeze-thaw cycles.

**Figure 4:** Variation law of unconfined compressive strength. (a) The relationship between freeze-thaw times of unconfined compressive strength. (b) Unconfined compressive strength-silt content relationship.

**Figure 5:** Intensity decay coefficient and freeze-thaw times.

**Figure 6:** Variation law of failure strain. (a) Relationship between failure strain and number of freeze-thaw cycles. (b) Relationship between failure strain and silt content.

**Table 1:** Density index of aeolian sand with cement alone.

Cement content (%)	Maximum dry density (g·cm^−3^)	Minimum dry density (g·cm^−3^)	Fill dry density (g·cm^−3^)	Relative density
0	1.70	1.49	1.63	0.70
3	1.76	1.48	1.69	0.78
5	1.79	1.47	1.72	0.81
7	1.81	1.46	1.74	0.83

## Data Availability

The data used to support the findings of this study are available from the corresponding author upon request.
